The article "An Intelligent and Reliable Hyperparameter Optimization Machine Learning Model for Early Heart Disease Assessment Using Imperative Risk Attributes" was retracted in 2023. Reasons: signs of a paper mill; suspected computer-generated content; unreliable results or conclusions; concerns about the data.

# An Intelligent and Reliable Hyperparameter Optimization Machine Learning Model for Early Heart Disease Assessment Using Imperative Risk Attributes

**DOI:** 10.1155/2022/9882288

**Published:** 2022-04-12

**Authors:** Syed Immamul Ansarullah, Syed Mohsin Saif, Syed Abdul Basit Andrabi, Sajadul Hassan Kumhar, Mudasir M. Kirmani, Dr. Pradeep Kumar

**Affiliations:** ^1^Lecturer at the Department of Computer Science, Govt. Degree College Sumbal, J&K, India; ^2^Research Coordinator at KWINTECH-R LABS (V), Kwintech-Rlabs(V), J&K, India; ^3^Research Scholar at the Department of Computer Science, Hyderabad, India; ^4^Research Scholar at the Department of Computer Science, Sehore, India; ^5^Assistant Professor at the Department of Computer Science, Division of Social Science, FoFy, SKAUST-Kashmir, Srinagar, India; ^6^Professor at the Department of Computer Science and Information Technology, MANUU, Hyderabad, India

## Abstract

Heart disease is a severe disorder, which inflicts an adverse burden on all societies and leads to prolonged suffering and disability. We developed a risk evaluation model based on visible low-cost significant noninvasive attributes using hyperparameter optimization of machine learning techniques. The multiple set of risk attributes is selected and ranked by the recursive feature elimination technique. The assigned rank and value to each attribute are validated and approved by the choice of medical domain experts. The enhancements of applying specific optimized techniques like decision tree, k-nearest neighbor, random forest, and support vector machine to the risk attributes are tested. Experimental results show that the optimized random forest risk model outperforms other models with the highest sensitivity, specificity, precision, accuracy, AUROC score, and minimum misclassification rate. We simulate the results with the prevailing research; they show that it can do better than the existing risk assessment models with exceptional predictive accuracy. The model is applicable in rural areas where people lack an adequate supply of primary healthcare services and encounter barriers to benefit from integrated elementary healthcare advances for initial prediction. Although this research develops a low-cost risk evaluation model, additional research is needed to understand newly identified discoveries about the disease.

## 1. Introduction

Heart disease is a growing socioeconomic and public health problem with significant mortality figures and disabilities [1]. The British Heart Foundation (BHF) and the Australian Bureau of Statistics (ABS) reported that heart disease causes 26% of all deaths in the United Kingdom and 33.7% of total deaths in Australia [2–6]. The Economic and Social Commission of Asia and the Pacific (ESCAP 2010) reports that 1/5th of Asian countries are afflicted with noncommunicable diseases like cancer, heart diseases, and chronic respiratory diseases [7].

The cost and mortality transformed heart disease into an epidemic worldwide. For example, the healthcare reports of the British, USA, and China show that heart disease per year in the UK is 9 billion pounds, 312.6 billion dollars in the USA, and 40 billion dollars in China. These reports show that the heart disease epidemic has a considerable effect on the world and is one of the dominant health and development challenges in terms of the human suffering they induce and the loss they impose on the socioeconomic foundation of countries [8–10].  Figure 1 shows the graphical demonstration of heart disease mortality rates across all countries through world map representation.

Different risk prediction tools are widely available to predict heart disease using clinical attributes obtained from multifaceted examinations in the medical lab but need prior blood sample investigation. In addition, there is no apparent known performance accuracy for them, which reduces their usability in other than medical settings. Considering the limitations of the existing risk tools and the social, economic, and public health effects of heart disease, we developed a heart disease risk assessment model that predicts the risk percentage with exceptional predictive accuracy at early stages [12, 13].

## 2. Literature Review

In recent times, researchers made influential contributions to heart disease prediction using various machine learning techniques.

Polat and Gunes proposed a novel system for the early prediction of cardiac disorders using the Artificial Immune Recognition System (AIRS) classifier with a fuzzy resource allocation mechanism [14]. They applied the K-NN-based weighting process to the heart disease dataset and scaled the weights in the range of 0 and 1 and then the fuzzy-AIRS algorithm was applied to the weighted heart disease dataset. Researchers obtain the heart disease dataset (containing 13 attributes and 270 instances) from the UCI Machine Learning Database. They achieved the highest classification accuracy after the value of *k* reached 15. The obtained classification accuracy result of the proposed system is 87%, and it is very promising concerning the other classification applications. The results strongly suggest that the K-NN-weighted preprocessing and fuzzy resource allocation mechanism of AIRS can assist in the prediction of cardiac arrhythmias.

Palaniappan and Awang developed a risk evaluation model using decision tree, neural network, and naive Bayes data mining techniques [15]. The developed model extracts interesting hidden patterns related to cardiac disorders and can answer detailed questions in which existing risk assessment tools fail. They developed a risk evaluation model on the .NET platform from the Cleveland heart disease database, containing 909 instances and 15 medical risk features. Researchers used the Data Mining Extension (DME) query language and functions to communicate with the model and checked its performance through a lift-chart and classification matrix. Experimental results show that the naive Bayes risk evaluation model outperforms neural network and decision tree models.

Tu et al. developed a predictive cardiac disorder risk model using bagging with naive Bayes, C4.5, and bagging with C4.5 classifiers on live datasets collected from patients with heart disease. The bagging algorithm neutralizes the instability of learning techniques by simulating the process using a given training set [16]. Instead of sampling a new training dataset each time, the original training data are modified by deleting some instances and replicating others. Researchers carried out three different experiments with the WEKA tool. Experiment 1 used the decision tree algorithm, experiment 2 used the bagging with the decision tree with a reduced error pruning option, and experiment 3 used the bagging with the naive Bayes algorithm. 10-fold cross-validation minimizes the bias produced by random sampling of each experiment's training and test data samples. Experimental results demonstrate that the precision, recall, and F-measure of bagging with naive Bayes optimal performance among the tested methods.

Adeli and Neshat developed a heart disease risk model using a fuzzy expert system [17]. The membership function of all the 11 input variables and 1 output variable utilizes an inference mechanism. Researchers use the Mamdani fuzzification and centroid method for the defuzzification process. The proposed system generated 44 rules and is best compared to the results of the other rule bases. Furthermore, they developed a validity degree (*k*) for each rule, and for the aggregation of rules, the maximum validity degree is calculated with *K* = max (*k*1, *K*2 … *k*44). Finally, the fuzzy expert diagnosis system shows that the system did relatively better than nonexperts.

Shouman et al. developed a classification model for early predicting heart disease patients using the decision tree technique. The multiple classifier voting techniques are integrated with different multi-interval discretization methods (equal frequency, chi-merge, equal width, and entropy) using different decision tree variants (Gini index, gain ratio, and information gain) [18]. The efficient heart disease decision rules are selected using the reduced error pruning technique. This model achieved the highest accuracy of 79.1% with equal width discretization without voting. After applying the voting technique, the equal frequency discretization gain ratio achieved the highest accuracy of 84.1%.

Shouman et al. developed a k-nearest neighbor risk evaluation model using the Cleveland heart disease dataset to detect cardiac disorder patients in advance with optimal accuracy [19]. They obtain the accuracy and the specificity of 97.4% and 99% when the value of *k* = 1 and 7, respectively. However, in this work, researchers discovered that applying the voting technique did not progress in precision even after estimating different parametric values of *k*.

Alizadehsani et al. applied C4.5 classification and bagging classifiers to investigate the lab and ECG data to identify the stenosis of each artery, left anterior descending (LAD), left circumflex (LCX), and right coronary artery (RCA), separately [20]. The random dataset of 303 instances is collected, and the feature selection method predicts the LAD stenosis accuracy. The Gini index and information gain select the essential features. Furthermore, the use of features selected based on information gain enhanced the accuracy of the LAD stenosis diagnosis to 79.54%. The results indicate that EF (ejection fraction), age, lymph, and HTN were among the ten most valuable features on the stenosis of all arteries.

Srinivas et al. proposed a new classifier by combining rough set theory with the fuzzy set for heart disease diagnosis [21]. Researchers generate fuzzy base rules using rough set theory, and the fuzzy classifier carries out the prediction. The proposed system uses MATLAB 7.11, and the presence of heart disease is identified by inputting the data to the fuzzy system. The classifier experiments on Cleveland, Hungarian, and Switzerland datasets, and results show that rough fuzzy classifier outperformed the previous approaches by achieving the accuracy of 80% on Switzerland's heart disease dataset and 42% on the Hungarian heart disease dataset.

Sumana and Santhanam proposed a hybrid risk model using best-first-search and feature selection techniques in a cascaded fashion [22]. Initially, they cluster the dataset using the k-means algorithm, and the correctly clustered samples are trained with 12 distinct classifiers to develop the final model using stratified 10-fold cross-validation. Next, they evaluate the model's performance using the WEKA tool on five other binary class medical datasets collected from the UCI machine learning repository to test the accuracy and time complexity of the classifiers. Experimental results show that the ensemble model enhanced the classification accuracy on five different medical datasets with all 12 classifiers.

Beena et al. selected the significant heart disease attributes by combining computerized feature selection methods and medical features to increase the prediction accuracy and decision-making for cardiac disorder diagnosis [23]. The default multiclass classification mode of the Cleveland heart disease dataset is converted into a binary classification form, and the sequential minimal optimization algorithm is applied to develop the risk model using the MATLAB tool. Experimental results show that the accuracy of the feature selection method increases by controlling the discrete features but the model time complexity increases.

Arabasadi et al. proposed a hybrid model based on clinical data without the need for invasive diagnostic methods. Researchers use feature selection techniques like the Gini index, weight by SVM, information gain, and principal component analysis (PCA) to train networks and modify weights to achieve minimum error [24]. They use the error back propagation algorithm in artificial neural network with MLP structure and sigmoid exponential function to build the heart disease model. The proposed risk model enhances the performance of neural network by increasing its initial weight using a genetic algorithm. The model achieves optimal accuracy, sensitivity, and specificity on the Z-Alizadeh Sani dataset, higher than the existing systems.

Dang et al. conducted a comprehensive survey of the latest IoT components, applications, and healthcare market trends [25]. They review the influence of cloud computing, ambient assisted living, big data, and wearables to determine how they help the sustainable development of IoT and cloud computing in the healthcare industry. Moreover, an in-depth review of IoT privacy and security issues, including potential threats, attack types, and security setups from a healthcare viewpoint, is conducted. Finally, this paper analyzes previous well-known security models to deal with security risks and provides trends, highlighted opportunities, and challenges for future IoT-based healthcare development. In addition, they do a comprehensive survey on cloud computing, particularly fog computing, including standard architectures and existing research on fog computing in healthcare applications.

Khan and Algarni proposed an Internet of Medical Things (IoMT) framework using modified salp swarm optimization (MSSO) and an adaptive neuro-fuzzy inference system (ANFIS) for early heart disease prediction [26]. The proposed MSSO-ANFIS technique gives higher values for precision, recall, F1-score, and accuracy and the lowest values for classification error compared with the existing metaheuristic and hybrid intelligent system methods. The proposed MSSO-ANFIS prediction model obtains an accuracy of 99.45 with a precision of 96.54, higher than the other approaches. However, different feature selection and optimization techniques need to be used to improve the model effectiveness of prediction.

Khan proposed a wearable IoT-enabled framework to evaluate heart disease using a modified deep convolutional neural network (MDCNN) [27]. The attached heart monitor device checks the blood pressure and electrocardiogram (ECG) of the patient. The MDCNN classifies the received sensor data into normal and abnormal. The proposed method shows that for the maximum number of records, the MDCNN achieves an accuracy of 98.2, which is better than existing classifiers. Furthermore, the proposed model shows better performance results than existing deep learning neural networks and logistic regression.

Khan et al. proposed a secure framework that uses the wearable sensor device which monitors blood pressure, body temperature, serum cholesterol, glucose level, etc. [28]. Patient authentication and sensor values transmit to the cloud server through the SHS-512 algorithm that uses substitution-Caeaser cipher and improved elliptical curve cryptography (IECC) encryption to ensure integrity. In improved ECC, a secret key is generated to enhance the system's security. In this way, the intricacy of the two phases is augmented. The computational cost of the scheme in the proposed framework is less than the existing schemes. The average correlation coefficient value is about 0.045, close to zero, showing the algorithm's strength. The intermediate encryption and decryption time are 1.032 and 1.004 s, respectively, lower than the ECC and RSA.

Morales-Sandoval et al. proposed a three-tier security model for wireless body area network (WBAN) systems suitable for e-health applications that provide security services in the entire data cycle [29]. An experimental evaluation determines the most appropriate cipher suites to ensure specific security services in an actual WBAN deployment. They observe that the cost of crypto-algorithms in terms of computational resources is acceptable. Specifically, the penalty in performance due to the computational processing of cryptographic layers can be tolerated by end users while still meeting the expected data rate of sensed data. Also, the proposed secure WBAN deployment design offers some degrees of freedom to provide different security levels (128, 192, and 256 bits) as desired. However, comparison with other methods is difficult due to the heterogeneous implementations of existing methods in terms of offered security services, device types, and security levels. In any case, the proposed security solution exhibits competitive performance in terms of execution time, memory, and energy consumption.

Ansarullah et al. developed an effective, low-cost, and reliable heart disease model using significant noninvasive risk attributes [30]. Feature selection techniques (extra tree classifier, gradient boosting classifier, random forest, recursive feature elimination, and XG boost classifier) and random forest, naive Bayes, decision tree, support vector machine, and K-nearest neighbor are applied to get significant risk attributes. Experimental results show that the random forest risk evaluation model outperforms other existing risk models with an admirable predictive accuracy of 85%.

The research activities and advancements have persistently enhanced in healthcare over the years.  Table 1 highlights the contributions, future work, and limitations of previous researches and discovers the possible potentials in heart disease risk evaluation using machine learning techniques.

## 3. Methodology

To build an intelligent and reliable hyperparameter optimization model for early heart disease assessment using imperative risk features, we used SEMMA methodology, consisting of five phases (Sample, Explore, Modify, Model, and Assess) as shown below in Figure 2. We collected primary heart disease data from heterogeneous data sources of Jammu & Kashmir consisting of 5776 patient records with 14 attributes. The Sample phase divides the dataset into a training, validation, and test dataset. The dataset is preprocessed and then split into 70% and 30% for training and testing purposes. After data division, the Explore phase visualizes the data and then the Modify phase is used to deal with the missing data. Once the data get complete from missing values and outliers, the Model phase implements the data mining and machine learning techniques. Finally, through the Assess phase of SEMMA, the test dataset is used to validate the derived model. We use the test dataset only once to avoid the model overfitting problem. In addition, we applied the cross-validation technique in model creation and refinement steps to evaluate the classification performance.

We applied recursive feature elimination, eliminating the least essential attributes per loop and removing the dependencies and collinearity among attributes [14]. The most critical risk attributes are marked as true and ranked 1, as shown in the below-given Table 2. We use multicollinearity and variance inflation factor (VIF) to identify the correlation and the strength of the correlation among the independent risk attributes [32, 33].

## 4. Optimized Risk Evaluation Model Development

We used Bayesian optimization and the single cross-validation technique to develop the risk evaluation model [34, 35]. The single cross-validation technique (Figure 3) divides the dataset into k-stratified sets. The decision tree, support vector machine, and k-nearest neighbor classifiers (excluding random forest algorithm) learn on the training dataset for every technique's solution. One part of the dataset validates the model, and the other half tests the model. The validation and test performances are measured through the model induced with the training dataset and the values of the hyperparameters found by the optimization technique. This process reiterates for all *k* combinations in single cross-validation. The average validation accuracy is then used as the fitness value, directing the search process. Finally, the individual with maximum validation accuracy is returned (with its hyperparameter value), and the technical performance is considered the average test accuracy of the individual.

## 5. Results and Discussion of Optimized Risk Models

### 5.1. Decision Tree Optimization Model

The most significant hyperparameters of the decision tree model are tuned to obtain optimal accuracy.

We validate them on the test data with careful evaluation to avoid overfitting [36–41]. After adjusting the hyperparameters of the decision tree model, we obtain the results given in Table 3. The permutations and combinations showed different results; however, we recorded only those combinations which provided the highest accuracy.

The optimized decision tree model has the true positive rate of 83.3%, which means the model can recognize the positive heart disease cases with an efficiency of 83.3%. Similarly, the model achieved a true negative rate of 80%, which means the model can recognize the nondiseased instances with 80% efficiency. As a result, the model reaches an accuracy of 81.85%, representing the overall accuracy in predicting both unhealthy and healthy heart disease cases which is 81.85%. Similarly, the precision is 82.94% which means the model has a low false-positive rate. The model's misclassification rate is 18%, and the AUROC score is 82%.

### 5.2. K-Nearest Neighbor Optimization Model

The primary hyperparameters of the K-NN model (the number of neighbors' *k* and the similarity function or the distance metric) are tuned to get the optimal results [30, 38, 39].

Table 4 describes the experimental results of the K-NN model. We use different permutations and combinations of the K-NN model to attain maximum accuracy. For example, when a metric attribute is Minkowski and the weight attribute is Uniform, the model's performance degrades 67%. The “best score” function checks the model's accuracy because the “best score” outputs the mean accuracy of the scores obtained through cross-validation. When hyperparameter combinations of the K-NN model are leaf size = 30, metric = city block, and weight = 13, the optimal results are achieved.

### 5.3. Support Vector Machine Optimization Model

The hyperparameters of SVM like [kernel, regularization, and gamma] are optimized, and we analyzed that the behavior of the developed SVM risk assessment model is extremely sensitive to the gamma hyperparameter [26–28].

Below, Table 5 shows the different accuracies achieved after tuning various hyperparameters of the SVM model. The hyperparameters (kernel and regularization) are adjusted with permutations and combinations to achieve optimal accuracy.

We observed that when kernel hyperparameter values are linear or sigmoid or sqrt, the time complexity of the risk model increases, and when parametric values are kernel = rbf, gamma = 0.1, and regularization = 1.0, we achieve the highest accuracy of 81%. In addition, we obtain the true positive rate of 80%, the true negative rate of 82%, an accuracy of 81%, the precision of 86%, the misclassification rate of 18%, and the AUROC curve value of 81%. We did not use the SVM model for the practical implementation because of its high time complexity, which causes an overfitting problem and results in disease misdiagnosis.

### 5.4. Random Forest Optimization Model

We explored and configured the most influential hyperparameters like N estimators, max depth, min sample split, min sample leaf, and max features of the random forest model [25, 29, 35].

The permutations and combinations of the optimized random forest model show different results recorded in Table 6. Experimental results show that when the hyperparameter combinations are as criterion = Gini, max depth = 50, max features = auto, and N estimators = 100, the highest accuracy of 87% is obtained. The performance results' true positive rate is 87%, the true negative rate is 84%, accuracy is 86%, precision is 86%, misclassification rate is 13%, and AUROC score is 86%.

## 6. Performance Comparison of Optimized Risk Models

This section describes the assessment and comparison of the hyperparameter optimization models. The performance of these models is testified through different model measures like true positive rate, true negative rate, accuracy, precision, error rate, and AUROC (described below Table 7). The results demonstrate that the optimized random forest model outclasses other developed risk models for these model performance measures. For example, the random forest model has a true positive rate of 87%, a true negative rate of 84%, an accuracy of 87%, a precision of 86%, AUROC of 87%, and the misclassification rate 13%.

Figure 4 shows the combined AUROC curves of different optimized risk evaluation models. For example, the random forest heart disease model has the highest AUROC score of 87%, which means the model can best differentiate among the diseased and nondiseased heart victims.

Furthermore, we verify the performance of the developed model with prevailing designs, which reveal that:

- The existing models only use the medical domain performance measures and do not consider the model performance measures like computational complexity, scalability, robustness, and comprehensibility. However, this risk evaluation model examines the both medical and model performance measures. As a result, the performance results show that the model has the high predictive capability and less computational complexity.
- Most heart disease models use invasive risk attributes; however, we develop a predictive risk model on noninvasive heart disease features.
- Most existing models use small secondary datasets for training, testing, and validation purposes, resulting in model overfitting; however, we use a substantial primary heart disease dataset to overcome biased diagnosis in this research.
- Most existing models lack generalization ability, but we developed an optimized model which adapts appropriately to new and previously unseen data.
- The existing risk models diagnose heart disease on complex and primarily derived rules, making the system slow and leading to wrong decisions; however, this risk model is simple with no complicated design. The simple rules extracted are used to create a chart as community screening tests to support healthcare experts in diagnosing heart disease patients.
- The developed risk evaluation model is innovative because it identifies the risk of heart disease based on noninvasive data features, thus supporting its application as a public screening test.

## 7. Conclusion

The existing risk tools predict heart disease using clinical attributes obtained from multifaceted examinations in the medical lab. This research developed an optimized risk evaluation model based on visible low-cost, noninvasive risk attributes. The recursive feature elimination and hyperparameter optimization methods like random forest, k-nearest neighbor, support vector machine, and decision tree algorithms are applied to discover an individual's degree of heart disease possessing specific risk attributes. We investigated the effect of different combined noninvasive features like age, sex, systolic bp, diastolic bp, BMI, and heredity to create a general level screening test to assess heart disease risk. We use out-of-sample testing to calculate the model performance measures. Experimental results show that the random forest model outperforms other models with the highest sensitivity, specificity, precision, accuracy, AUROC score, and minimum misclassification rate. We simulate the accomplished outcomes with the prevailing research; the results obtained are more excellent than published values in the literature to the best of our perception. This model will support medical practitioners and provide victims with a message about the possible existence of risk even before they visit a clinic or do exorbitant health inspections. Furthermore, this model is applicable where people lack the facilities of integrated primary medical care technologies for untimely prediction and cure.

## 8. Future Work

- We would enhance the research work by adding other noninvasive attributes (socioeconomic level, depression level, and ethnicity) to the performance of different data mining methods.
- We will identify the significance of controlled noninvasive attributes such as weight and smoking in different age and sex groups in heart disease risk estimation.
- We would enhance the research by using heterogeneous real-world datasets with different attributes, diverse population groups, and many records.
- We will develop a one-size-fits-all heart disease risk model using data mining techniques to prescribe a treatment plan for the disease successfully.

## Figures and Tables

**Figure 1:** World map showing the global distribution of heart disease mortality rates [11].

**Figure 2:** Description of SEMMA data mining methodology [31].

**Figure 3:** Showing single cross-validation technique for hyperparameter optimization.

**Figure 4:** Combined AUROC of the optimized risk evaluation models.

**Table 1:** List of contributions from previous surveys on heart disease prediction using machine learning techniques.

Ref	Year	Dataset	Results	Contribution	Future work	Limitations
[14]	2007	UCI heart disease dataset contains 13 attributes and 270 instances	Weighted K-NN/87% accuracy	Proposed a cardiac arrhythmia model using K-NN-weighted preprocessing and fuzzy allocation mechanism of artificial immune recognition system	To enhance the model by applying SVM, decision tree, and hybrid techniques	(i) This model identifies only a type of heart disease
						(ii) The small dataset size is not ideal for stable performance because it results in biased measurements
[15]	2008	Cleveland heart disease dataset has 909 instances and 15 medical risk features	Naive Bayes/95% accuracy	They developed a risk model using decision tree, neural network, and naive Bayes algorithms	To improve model performance by training on massive data	(i) Small dataset with limited instances
						(ii) Overfitting problems occur in a small dataset, leading to poor performance with the test data
[16]	2009	Researchers obtain live datasets from patients with heart disease	Bagging with naive Bayes/84.1% accuracy	Developed risk model using C4.5, bagging with naive Bayes, and bagging with C4.5	To develop a robust heart disease risk model using python or R	Weka handles small datasets, and whenever a dataset is bigger than a few megabytes, an OutOfMemoryError occurs
[17]	2010	UCI data repository	The accuracy of the developed model is 82%	(i) Develop fuzzy expert risk model	Build an ensemble model because that will result in a robust and optimal model and increase the model's efficiency	Derived rules from the cardiovascular disease dataset are complex and large, making the system slow and making wrong decisions
				(ii) It generated 44 rules compared with the results of other rule bases.		
[18]	2011	Cleveland heart disease dataset has 909 instances and 15 medical risk features	The accuracy of 79.1% with voting and 84.1% without voting is achieved	(i) Develop a classification model using the decision tree	To develop a risk evaluation model using hybrid classification techniques for optimal results	The developed heart disease evaluation models lack generalization ability
				(ii) Heart disease rules are generated using reduced error pruning		
[19]	2012	Cleveland heart disease dataset	K-NN with the accuracy of 97%	They develop the K-NN model for the early prediction of heart disease	To work on a primary heart disease dataset with considerable volume size	Applying the voting technique did not progress in precision even after estimating different parametric values of k
[20]	2013	The random dataset of 303 instances is collected	The accuracy of the LAD stenosis is 79.54%	(i) They apply C4.5 and bagging to check the lab and ECG data	To work on a primary heart disease dataset with massive instances using hybrid learning techniques	The model uses invasive risk features, making it difficult for general users and limiting its usage to the medical domain
				(ii) The Gini index and information gain select the essential features		
[21]	2014	Used Cleveland, Hungarian, and Switzerland datasets	80% and 42% accuracies on Switzerland and Hungarian heart disease datasets, respectively	(i)Proposed a model by combining rough set theory with the fuzzy set	To develop a risk evaluation model with less computational complexity and high predictive capability	They use medical domain performance measures and do not test the model measures (computational complexity, scalability, robustness, and comprehensibility)
				(ii) Generate fuzzy base rules using the rough set approach and the fuzzy classifier.		
[22]	2015	Five binary class medical datasets collected from the UCI repository	Optimal results	Initially, the k-means algorithm is used for clustering and then 12 distinct classifiers are used to create the final model using stratified 10-fold cross-validation	To develop a risk model with the best generalization ability and less computational complexity	(i) The developed risk model is complex and takes more computational time
						(ii) Used Weka tool that handles small datasets, and an OutOfMemoryError occurs on a vast dataset
[23]	2016	Cleveland heart disease dataset	Accuracy increases by controlling the discrete features using feature selection techniques	Sequential minimal optimization algorithm is applied to develop the risk model using the MATLAB tool	To extend the model by using real-time datasets to get an accurate diagnosis in advance	(i) The model time complexity is high
						(ii) Overfitting problems occur in a small dataset, leading to poor performance with the test data
[24]	2017	Used Z-Alizadeh sani heart disease dataset	The accuracy, sensitivity, and specificity are 84%, 85%, and 89%	Proposed a hybrid model that uses the error back propagation algorithm in ANN with MLP structure and sigmoid exponential function	Develop a one-size-fits-all heart disease model to successfully prescribe a treatment plan for the disease	The error generated by the hidden neurons on output nodes degrades the neural network's logic potential, resulting in wrong prediction and decision-making
[31]	2019	Review paper	Analyze security models, check trends, and highlight opportunities and challenges for future IoT-based healthcare development	(i) Review latest IoT components, applications, and healthcare market trends	Will address the challenges that prevent the development of IoT and cloud computing in healthcare, such as data security, system development processes, and business models	They did not review IoT privacy and security issues like potential threats, attack types, and security setups
				(ii) Analyze the influence of cloud computing, big data, and wearables to determine how they help the sustainable development of IoT and cloud computing in the healthcare industry		
[14]	2020	Unknown	MSSO-ANFIS/accuracy = 99.4 and precision = 96.54	Propose an Internet of Medical Things framework using modified salp swarm optimization and an adaptive neuro-fuzzy inference system for heart disease prediction	Researchers will use different feature selection and optimization techniques to improve the model effectiveness of prediction	The developed heart disease prediction model is complex and expensive because of medical attribute examination and IoT use
[32]	2020	Live dataset	MDCNN/accuracy = 98.2	Propose a wearable IoT-enabled framework to evaluate heart disease using a modified deep convolutional neural network (MDCNN)	(i) To increase the model's performance using other feature selection and optimization techniques	The developed risk model is complex and expensive because of medical attribute examinations and IoT use
				The MDCNN classifies the received sensor data into normal and abnormal	(ii) To train the model with fully wearable devices available in the market	
[33]	2020	Live dataset	Avg. correlation coefficient is 0.045, encryption time = 1.032S, and decryption time = 1.004 S	Proposed a secure framework that uses the wearable sensor device which monitors blood pressure, body temperature, serum cholesterol, glucose level, etc	To extend this work, such as capturing the data from the wearable sensors and performing real-time analysis	The developed framework is complex because of the use of IoT components
[34]	2021	Wireless body area networks (WBAN) framework	Execution time, memory, and energy consumption of the developed WBAN are optimal	Propose a three-tier security model for wireless body area networks (WBAN) systems that is suitable for e-health applications	To incorporate the security solutions and concentrate on competitive execution time, memory, and energy consumption	(i) They used lightweight cryptography instead of robust crypto-algorithms
						(ii) A complete comparison with other methods is difficult due to security services, device types, and security levels.
[35]	2022	Primary heart disease dataset consisting of 5776 records	Random forest/85% accuracy	Develop an effective, low-cost, reliable risk evaluation model using significant noninvasive risk attributes	(i) To enhance the risk model by adding other noninvasive features	The risk model is developed on a specific population, hence narrowing its application
					(ii) To investigate deep learning and study the significance of other controlled features on different age and sex groups	

**Table 2:** Risk attribute ranking using recursive feature elimination technique.

Risk attributes	Values	Ranking	VIF factor
Age	True	1	1.1
Sex	False	2	1.4
Height	True	1	1.1
Weight	True	1	1.1
Systolic BP	True	1	1.3
Diastolic BP	True	1	1.1
Hereditary	True	1	1.2
Unhealthy diet	True	1	1.1
Physical activity	True	1	1.2
Alcohol consumption	False	2	1.5
Smoking	False	2	1.7
Socioeconomic level	False	1	1.3

**Table 3:** Showing experimental results of the optimized decision tree model.

Max depth	Min samples split	Min samples leaf	Max features	Criterion	Accuracy
10	18	15	Auto	Entropy	81%
15	25	12	Auto	Gini	82%
18	11	10	Sqrt	Gini	72%
20	15	20	Sqrt	Gini	83%
25	10	50	Auto	Entropy	71%
30	12	30	Auto	Entropy	74%
35	22	25	Sqrt	Entropy	75%
40	8	14	Sqrt	Gini	78%
45	5	16	Auto	Entropy	73%
50	14	0	Auto	Gini	78%
70	17	18	Auto	Entropy	75%
80	13	0	Auto	Entropy	84%
100	20	0	Sqrt	Entropy	84%

**Table 4:** Showing experimental results of the optimized K-NN model.

Leaf size	Metric	Neighbors	Weights	Accuracy
5	Euclidean	5	Distance	82%
10	Minkowski	11	Uniform	67%
30	City block	13	Distance	85%
25	Euclidean	9	Distance	70%
15	Minkowski	7	Uniform	72%
20	City block	11	Uniform	68%
12	Euclidean	15	Distance	75%
16	Minkowski	13	Uniform	77%
18	Minkowski	7	Uniform	80%
28	Euclidean	9	Distance	82%

**Table 5:** Showing experimental results of the optimized SVM model.

Kernel	Gamma	Regularization	Accuracy
Linear	0.001	0.11	71%
Sigmoid	0.1	1.0	70%
Sqrt	0.00001	0.001	68%
Rbf	0.1	1.0	81%
Linear	0.001	0.001	72%
Rbf	0.0001	0.1	80%
Linear	0.01	0.10	73%
Rbf	0.0011	0.0001	78%
Sqrt	0.0001	0.010	75%
Sqrt	0.1	0.11	76%
Sigmoid	0.01	1.0	74%
Linear	0.0001	1.0	71%
Sigmoid	0.010	0.11	77%
Rbf	0.11	0.0001	69%
Sqrt	0.10	0.001	73%

**Table 6:** Shows the experimental results of the optimized random forest model.

Criterion	Max depth	Max features	*N* Estimators	Min samples leaf	Accuracy
Gini	70	0	0	0	85%
Entropy	60	Auto	0	0	86%
Gini	50	Auto	100	0	87%
Entropy	80	Auto	100	100	73%
Gini	100	Auto	100	50	76%
Entropy	30	0	80	60	80%
Gini	40	0	90	40	78%
Gini	25	Auto	70	30	75%
Entropy	20	Auto	40	25	82%
Entropy	35	Auto	30	20	81%
Gini	45	0	60	35	80%

**Table 7:** Showing performance measures of the developed optimized heart disease models.

	Performance measures of the models					
Models	TPR	TNR	Accuracy	Precision	Error rate	AUROC

Decision tree	83%	80%	82%	82%	5%	82%
K-NN	87%	81%	84%	83%	15%	85%
SVM	80%	82%	82%	86%	18%	82%
Random forest	87%	84%	87%	86%	13%	87%

## Data Availability

The heart disease risk data used to support the findings of this study are included within the supplementary information file.

## Supplementary Materials

Supplementary Materials The heart disease risk data used to support the findings of this study are included within the supplementary information file. Data of the heart disease risk are in the supplementary section.

## References

[1] Gaziano T. A., Bitton A., Anand S., Abrahams-Gessel S., Murphy A., Murphy A. (2010). Growing epidemic of coronary heart disease in low- and middle-income countries. *Current Problems in Cardiology*.

[2] Tran J., Norton R., Conrad N. (2018). Patterns and temporal trends of comorbidity among adult patients with incident cardiovascular disease in the UK between 2000 and 2014: a population-based cohort study. *PLoS Medicine*.

[3] Australian Bureau of Statistics (2013). *Australian Health Survey: Biomedical Results for Chronic Diseases, 2011–12. ABS Cat. No. 4364.0.55.005*.

[4] Australian Bureau of Statistics (2015). *National Health Survey: First Results, 2014–15. ABS Cat. No. 4364.0.55.001*.

[5] Australian Bureau of Statistics (2016). *Causes of Death, Australia, 2015. ABS Cat. No. 3303.0*.

[6] Australian Institute of Health and Welfare (2009). *Impact of Falling Cardiovascular Disease Death Rates: Deaths Delayed and Years of Life Extended. Bulletin No. 70. Cat. No. AUS 113*.

[7] Song P., Gupta A., Goon I. Y. (2021). Data resource profile: Understanding the patterns and determinants of health in South Asians-the South Asia Biobank. *International Journal of Epidemiology*.

[8] Virani S. S., Alonso A., Benjamin E. J. (2020). American heart Association Council on Epidemiology and prevention Statistics Committee and Stroke Statistics Subcommittee. Heart disease and Stroke Statistics-2020 Update: a report from the American heart Association. *Circulation*.

[9] Heidenreich P. A., Albert N. M., Allen L. A. (2013). Forecasting the Impact of heart Failure in the United States. *Circulation: Heart Failure*.

[10] Rti International (2017). Cardiovascular disease costs will exceed $1 trillion by 2035: Nearly half of Americans will develop pre-existing cardiovascular disease conditions, analysis shows. *Science Daily*.

[11] Bank I. E., Timmers L., Gijsberts C. M. (2015). The diagnostic and prognostic potential of plasma extracellular vesicles for cardiovascular disease. *Expert Review of Molecular Diagnostics*.

[12] Ng R., Sutradhar R., Kornas K. (2020). Development and validation of the chronic disease population risk tool (CDPoRT) to predict Incidence of adult chronic disease. *JAMA Network Open*.

[13] GBD Risk Factors Collaborators (2015). Global, regional, and national comparative risk assessment of 79 behavioral, environmental and occupational, and metabolic risks or clusters of risks, 1990–2015: a systematic analysis for the Global Burden of Disease Study. *The Lancet*.

[14] Polat K., Güneş S. (2007). A hybrid approach to medical decision support systems: combining feature selection, fuzzy weighted pre-processing and AIRS. *Computer Methods and Programs in Biomedicine*.

[15] Palaniappan S., Awang R. (2008). Intelligent heart disease prediction system using data mining techniques. *IEEE/ACS Int. Conf. Comput. Syst. Appl*.

[16] Tu My C., Shin D., Shin D. K. Effective diagnosis of heart disease through bagging approach.

[17] Ali A., Neshat M. (2010). A fuzzy expert system for heart disease diagnosis. *Proceedings of the International MultiConference of Engineers and computer scientists*.

[18] Shouman M., Turner T., Stocker R. (2011). Using decision tree for diagnosing heart disease patients. *Proc. Proceedings of the Ninth Australasian Data Mining Conference, Ballarat, Australia*.

[19] Shouman M., Turner T., Stocker R. Using data mining techniques in heart disease diagnosis and treatment.

[20] Alizadehsani R., Habibi J., Hosseini M. J. (2013). A data mining approach for diagnosis of coronary artery disease. *Computer Methods and Programs in Biomedicine*.

[21] Srinivas K., Rao G. R., Govardhan A. Rough-fuzzy classifier: a system to predict the heart disease by Blending two different set Theories. *Arabian Journal for Science and Engineering*.

[22] Sumana B. V., Santhanam T. Prediction of diseases by cascading clustering and classification.

[23] Bethel B. G. N., Rajinikanth T. V., Raju V. S. (2016). A Knowledge-driven approach for efficient analysis of heart disease dataset. *International Journal of Computer Applications*.

[24] Arabasadi Z., Alizadehsani R., Roshanzamir M., Moosaei H., Yarifard A. A. (2017). Computer aided decision making for heart disease detection using hybrid neural network-Genetic algorithm. *Computer Methods and Programs in Biomedicine*.

[25] Dang L. M., Piran M. J., Han D., Min K., Moon H. (2019). A survey on Internet of Things and cloud computing for healthcare. *Electronics*.

[26] Khan M. A., Algarni, F. (2020). A healthcare monitoring system for the diagnosis of heart disease in the IoMT cloud Journal of Healthcare Engineering 11 Environment using MSSO-ANFIS. *IEEE Access*.

[27] Khan M. A. (2020). An IoT framework for heart disease prediction based on MDCNN classifier. *IEEE Access*.

[28] Khan M. A., Quasim M. T., Alghamdi N. S., Khan M. Y. (2020). A secure framework for authentication and encryption using improved ECC for IoT-based medical sensor data. *IEEE Access*.

[29] Morales-Sandoval M., De-La-Parra-Aguirre R., Galeana-Zapién H., Galaviz-Mosqueda A. (2020). A three-tier approach for Lightweight data security of body area networks in E-health applications. *Access IEEE*.

[30] Ansarullah S. I., Saif S. M., Kumar P., Kirmani M. M. (2022). Significance of visible non-invasive risk attributes for the initial prediction of heart disease using different machine learning techniques. *Computational Intelligence and Neuroscience*.

[31] SAS Enterprise Miner – SEMMA (2008). SAS Institute. http://www.sas.com/technologies/analytics/datamining/miner/semma.html.

[32] Rezaee M., Putrenko I., Takeh A., Ganna A., Ingelsson E. (2020). Development and validation of risk prediction models for multiple cardiovascular diseases and Type 2 diabetes. *PLoS one*.

[33] Wu J., Chen X.-Y., Zhang H., Xiong Li-D., Lei H., Deng Si-H. (2019). Hyperparameter optimization for machine learning models based on Bayesian optimization. *Journal of Electronic Science and Technology*.

[34] Mantovani R. G., Horvath T., Cerri R., Vanschoren J., de Carvalho A. C. P. L. F. Hyper-Parameter tuning of a decision tree Induction algorithm.

[35] Tabrez Quasim M., Algarni F., Radwan A. A. E., M Alshmrani G. M. A Blockchain-based secured healthcare framework.

[36] Feurer M., Hutter F. (2019). Hyperparameter optimization. *Automated Machine Learning*.

[37] Jiang W. e. i., Siddiqui S. (2020). Hyper-parameter optimization for support vector machines using stochastic gradient descent and dual coordinate descent. *EURO Journal on Computational Optimization*.

[38] Elgeldawi E., Sayed A., Galal A. R., Zaki A. M. (2021). Hyperparameter tuning for machine learning algorithms used for Arabic Sentiment analysis. *Informatics*.

[39] Kumhar S. H., Kirmani M. M., Sheetlani J., Hassan M. (2021). Word embedding generation for Urdu language using Word2vec model. *Materials Today: Proceedings*.

[40] Kumhar S. H., Kirmani M. M., Sheetlani J., Hassan M. (2020). Word embedding generation methods and tools: a critical review. *International Journal of Innovative Research in Computer and Communication Engineering*.

[41] Ansarullah, Immamul S., Kumar P. (2019). A systematic literature review on cardiovascular disorder identification using knowledge mining and machine learning method. *International Journal of Recent Technology and Engineering*.

